The article "Investigating IT Faculty Resistance to Learning Management System Adoption Using Latent Variables in an Acceptance Technology Model" was published in 2015. Journal: ScientificWorldJournal.

# Investigating IT Faculty Resistance to Learning Management System Adoption Using Latent Variables in an Acceptance Technology Model

**DOI:** 10.1155/2015/375651

**Published:** 2015-09-30

**Authors:** Fatiha Bousbahi, Muna Saleh Alrazgan

**Affiliations:** Information Technology Department, College of Computer and Information Sciences, King Saud University, P.O. Box 22452, Riyadh 11495, Saudi Arabia

## Abstract

To enhance instruction in higher education, many universities in the Middle East have chosen to introduce learning management systems (LMS) to their institutions. However, this new educational technology is not being used at its full potential and faces resistance from faculty members. To investigate this phenomenon, we conducted an empirical research study to uncover factors influencing faculty members' acceptance of LMS. Thus, in the Fall semester of 2014, Information Technology faculty members were surveyed to better understand their perceptions of the incorporation of LMS into their courses. The results showed that personal factors such as motivation, load anxiety, and organizational support play important roles in the perception of the usefulness of LMS among IT faculty members. These findings suggest adding these constructs in order to extend the Technology acceptance model (TAM) for LMS acceptance, which can help stakeholders of the university to implement the use of this system. This may assist in planning and evaluating the use of e-learning.

## 1. Introduction

The impact of information and communication technologies (ICT) has influenced teaching and learning strategies [1]; specifically, it has enabled learning by electronic media (e-learning). Consequently, there has been an increasing demand for distance and online learning. Additionally, development of the e-learning platform has changed education from teacher centered to student-centered by enabling teachers mentoring learning rather than merely delivering information. Instructors need to improve the system of teaching and learning by providing useful resources and activities for students through the use of technology. Therefore, teachers need to adopt these new technologies and use them wisely to deliver material to students. For example, faculty members should utilize ICT by implementing the use of learning management system.

A learning management system (LMS) is a software application used to deliver online material and training programs to students while tracking their progress and generating related reports [2]. An LMS increases independence through the use of technology while simultaneously promoting interaction and collaboration between students and teaching staff outside the classroom [1]. One available tool in an LMS is an online discussion forum that enhances the foundation of the class for the students by enabling asynchronous communication and facilitating problem solving. LMS programs have often been promoted as an efficient means to deliver high-quality learning for students by providing constant access to learning materials, while permitting efficient course management for teachers. While there are many available LMS programs, the most popular is Blackboard, which will be used in our study.

The article "Investigating IT Faculty Resistance to Learning Management System Adoption Using Latent Variables in an Acceptance Technology Model" was published in 2015. Journal: ScientificWorldJournal.

Recently, the Ministry of Education in Saudi Arabia approved e-learning as a component of its national plan. This plan calls for the adoption of e-learning, distance learning, and blended learning in higher education [3]. One of the plan achievements has been the establishment of the Saudi Electronic University in 2011. This institution offers both graduate and undergraduate programs [4]. Along the same lines, various universities around the kingdom have established the deanship of e-learning and hired dedicated staff to support blended learning and the adoption of LMS in university courses. This e-learning deanship has offered training courses related to how to use tools to design digital courses for interested faculty members. Currently, however, LMS programs tend to be used as mere vaults to house and disperse course data rather than to improve student learning outcomes. It could be the case that instructors lack experience with computer-based interactions like facilitating asynchronous discussions groups or administering online quizzes [2]. It is useful to inquire whether this holds true for instructors who are teaching Information Technology courses, as well.

While numerous studies focused on usage intention and behavior toward LMS acceptance, little research has highlighted the impact of external variables on LMS usage as suggested by [5–7]. Therefore, it is necessary to conduct research that investigates intensively to uncover factors influencing LMS (e-learning) acceptance in teaching. However, minimal research has been conducted in Saudi Arabia to empirically determine the relationship of faculty members and LMS use with personal factors such as motivation, anxiety, LMS perceived usefulness (PU), LMS perceived ease of use (PEOU), and organizational support.

In the present study, we focus on understanding the antecedents of LMS usage in higher education at King Saud University, especially among Information Technology faculty members, and we assess how the factors of interest interact with each other.

The organization of this paper is as follows: first, we state the research problem and objectives along with research hypotheses related to the latent variables of acceptance of the technology model. Subsequently, a survey of the proposed acceptance models is presented in Literature Review. Next, we establish the layout of the research design and methodology consisting of study setting, data collection instruments, design of the study process, and data analysis procedures. We then present the findings of this research and provide meaningful analysis based on faculty members' comments as well as on regression models. Finally, we conclude our paper and provide some suggestions for future work.

The article "Investigating IT Faculty Resistance to Learning Management System Adoption Using Latent Variables in an Acceptance Technology Model" was published in 2015. Journal: ScientificWorldJournal.

## 2. Research Problem

At KSU LMS has been adapted for several years; some faculty members have embraced it while others have not. Among the faculties who resisted the acceptance of LMS are the majority of Information Technology (IT) faculties. Presently quarter or less of the IT faculty members use LMS (Blackboard) in their teaching. They also have experienced low motivation toward training and using this tool in their daily classroom activities. The problem under investigation revolves around understanding reasons for the lower rate of usage of LMS for teaching and learning within the IT Department. The level of acceptance and the causes of resistance had to be identified to provide insights to encourage the successful implementation of LMS (Blackboard) as e-learning platform. According to previous studies [6, 8–11] motivation, computer anxiety, and organizational support were all determinants of PEOU and PU [6]. Previous research found that computer anxiety influences users PEOU of an information system. For example, Teo (2011) in [12] found that female had a higher level of computer anxiety compared to male. Although similar attempts have been done in previous research, we did not find any studies which examined these specific factors simultaneously as external variables influencing LMS (even IS) acceptance as postulated in TAM. We hope this study will provide additional understanding of anxiety, motivation, organizational support, PEOU, and PU relationship and their role in LMS usage.

## 3. Research Objectives

This study will adopt part of the technology acceptance model (TAM) [13] to study the variables that most significantly affect the acceptance of LMS among IT faculty members. The objective of our study is to analyze the relationship of faculty usage of LMS while offering blended-learning courses. The selected constructs are motivation, load anxiety, perceived usefulness, perceived ease of use, organizational support, and actual use of LMS.  Table 1 shows the different variables in this study, as the first column lists the variables, the second column indicates the number of items (questions) used to measure each of the variables and shows the theoretical support for each of them, and the third column provides reference to previous studies.

The article "Investigating IT Faculty Resistance to Learning Management System Adoption Using Latent Variables in an Acceptance Technology Model" was published in 2015. Journal: ScientificWorldJournal.

## 4. Research Hypotheses

The purpose of our study was to investigate the correspondence between faculty usage of LMS and the following variables: motivation, load anxiety, support, perceived usefulness, and perceived ease of use. The following question was asked: What are the relationships between these external variables and faculty attitudes related to the adoption of e-learning technologies? From this research question, we have derived the following hypotheses:

(H1) An increase of positive organizational support, perceived usefulness, perceived ease of use, and reduced load anxiety toward Blackboard will lead to a statistically significant increase in the motivation variable.
(H2) An increase of positive motivation, organizational support, perceived usefulness, and perceived ease of use toward Blackboard will lead to a statistically significant reduction in load anxiety among IT faculty.
(H3) An increase of positive motivation, perceived usefulness, reduced load anxiety, and perceived ease of use toward Blackboard will lead to a statistically significant increase in organizational support.
(H4) An increase of positive motivation, organizational support, reduced load anxiety, and perceived ease of use toward Blackboard will lead to a statistically significant increase in perceived usefulness.

## 5. Literature Review

The literature addressing the acceptance of technology has witnessed a significant increase of research in the last decade. This research was mainly conducted to understand technology acceptance in the industrial environment. In [15], technology acceptance was defined as a user's willingness to employ technology for the tasks it is designed to support. Several case studies were conducted to identify and explain factors influencing the adoption of technology in order to minimize resistance or rejection [12]. Furthermore, technology is an essential part of e-learning.

E-learning describes a technology-rich learning environment. It has been discussed in much research as a tool for improving student learning processes and enhancing teaching practices. Learning management systems are considered to be essential tools to facilitate e-learning and are being employed by numerous universities to facilitate and expand learning opportunities. Nevertheless, this technology is often not used to its full potential.

Teachers are ultimately responsible for the final decision to either use or avoid technology. To understand why teachers accept or reject e-learning, one must understand why teachers accept or reject technology [12].

The article "Investigating IT Faculty Resistance to Learning Management System Adoption Using Latent Variables in an Acceptance Technology Model" was published in 2015. Journal: ScientificWorldJournal.

Many models designed to evaluate user acceptance are cited in the literature; an overview of these studies is presented in [5]. The technology acceptance model (TAM) is one of the most popular models used to examine users' acceptance of technology [13]. It has its roots in the Theory of Action (TRA) model designed by Ajzen and Fishbein [16]. According to TAM, the use of an information system (IS) depends on the intent of a person to use this system. This intention is determined by the attitude of the individual relative to the IS. This attitude is itself influenced by the perceived usefulness and the perceived ease of use, which are both determinants of the use of IS [5]. TAM replaces many of the TRA behavior constructs with two factors to predict user acceptance: perceived ease of use (PEOU) (“the degree to which a person believes that using a particular system would be free of effort”) and perceived usefulness (PU) (“the degree to which a person believes that using a particular system would enhance his/her job performance”) [5]. The overall approach of TAM is predictive attempting to identify the constructs impacting users' intentions to use technology. These two variables were validated by Davis [5] to be fundamental determinants of user acceptance. Numerous empirical studies have concluded that TAM is the most simple model, the most easy to apply, and the most robust to explain IT/IS usage in business contexts [6, 7, 17]. Nevertheless, the external variables that are likely be much more influential in a particular context remain to be identified, as stated by Davis in [5]. He suggested that further studies are needed to extend TAM with additional variables. The TAM is presented in Figure 1.

Thus, the TAM, besides having been validated several times by various researchers, was also subjected to various improvements and adaptations, beginning with its author. In a subsequent project, Venkatesh and Davis [8] developed an extension of TAM named TAM2. TAM2 tends to identify the elements that influence the perceived usefulness and intentions to use technology by adding two constructs: social influence and cognitive instrumental processes. The first construct refers to volunteering, subjective norms, and image; the second refers to job relevance, output quality, and demonstration of tangible results. The model was validated with a variance of 40%–60% for the perceived usefulness and 34%–52% variance for the intended use.

Additionally, in [7], the authors reviewed eight models related to acceptance of technology. Their study had led to the birth of a new extension of TAM: Unified Theory of Acceptance and Use of Technology, or UTAUT. In this extension, the construct of attitude is not taken into account. UTAUT uses three determinants for intention use, performance expectancy, effort expectancy, and social influences, and one determinant, facilitating behavioral conditions for usage. The empirical results of this model showed a high-explained variance of approximately 70%. However, in their study's conclusion, the authors recommended future work to seek new constructs to explain the intention of use.

The article "Investigating IT Faculty Resistance to Learning Management System Adoption Using Latent Variables in an Acceptance Technology Model" was published in 2015. Journal: ScientificWorldJournal.

Along the same lines, the authors in [6] examined the influence of contextual specificity when describing technology acceptance. Based on social cognitive theory, they added six independent variables to the technology acceptance model (TAM), computer anxiety, prior experience, organizational support, task structure, and system quality, as well as one intervening variable (computer efficacy). The authors tested the extended model (Figure 2) using a mail survey and results were tabulated using partial least squares analysis. The results showed that system usage was strongly influenced by computer anxiety, prior experience, organizational support, task structure, system quality, and perceived usefulness. In addition, perceived usefulness was the strongest mediator in determining system usage. The model was tested with all of the relations between the constructs in a context of PC usage and satisfied results.

While different versions of TAM have focused on utility, usability, and acceptability of IS in business contexts, other authors [12, 18–20] have applied these models in education, taking into account the pedagogical usefulness factor. These studies will be explained as follows.

One interesting study in [20] used the technology acceptance model (TAM) constructs of usefulness and ease of use to assess university students' acceptance of course websites as an effective learning tool. A survey instrument was distributed to 450 undergraduate students, and a total of 403 usable responses were obtained. The author implemented exploratory and confirmatory factor analyses using structural equation modeling techniques. This was subsequently used to fit and validate the Course Website Acceptance Model (CWAM) designed for this study. Results obtained through the CWAM indicated good fit to the data. Course website usefulness and ease of use proved to be key determinants of the acceptance and usage of course websites as an effective and efficient learning technology. The causal relationships between the constructs considered by the CWAM were well supported, accounting for 83% of the total variance in the course website acceptance and usage.

Furthermore, another useful study [21] analyzed TAM in higher education to understand students' behavioral intention to use e-learning. The author tested the relationship of students' intention to use e-learning with multiple constructs including their attitude, perceived usefulness, perceived ease of use, self-efficacy of e-learning, subjective norm, and system accessibility. He concluded that TAM is a good theoretical tool to understand users' acceptance of e-learning and found that learning self-efficacy considered as an intrinsic motivational factor was the most important construct, followed by subjective norm in clarifying the causal process in the model.

The article "Investigating IT Faculty Resistance to Learning Management System Adoption Using Latent Variables in an Acceptance Technology Model" was published in 2015. Journal: ScientificWorldJournal.

More recently, researchers have focused on faculty acceptance of using web-based e-learning rather than traditional classroom formats. They relied on the technology acceptance model (TAM) as a basis to understand the adoption of e-learning in higher education. We will report some of these studies in the following section.

In [19], the author remarked that teachers are not using technology as much as expected in American schools and addressed two questions in his dissertation: “(1) how often and to what extent do secondary teachers use web-based e-learning technology to support student learning; (2) What factors influence teacher acceptance or rejection of technology in their teaching.” In his study, the Unified Theory of Acceptance and Use of Technology (UTAUT) model was adopted and used as a theoretical framework to determine the teachers' actual use of e-learning. A survey was distributed to teachers in five northeastern Pennsylvania high schools, and interviews were conducted by the author. A total of 151 teachers responded to the survey. The author employed a correlational mixed-method to examine the influence that several independent variables including performance expectancy, effort expectancy, social influence, and facilitating conditions have on secondary school teachers' acceptance of e-learning technology. The results of this study revealed that performance expectancy was the most dominant factor in determining teachers' acceptance and use of e-learning, in addition to other factors such as effort expectancy and facilitating conditions, which were also found to play a role in acceptance.

A seminal study in this area is the work presented in [9]. The author had proposed a new model: the motivation and acceptance model (MAM), which is a combination of the technology acceptance model (TAM) and the Commitment and Necessary Effort (CANE) model. The author adopted in this MAM the following variables: perceived usefulness, perceived organizational support, perceived ease of use, and faculty attitude. The aim of this study was to investigate faculty perception and their use of a new software program called LiveText. The author had tested his model among the faculty of Southeastern University using regression analysis. The findings suggested that attitude had an impact on the usage of new software, and, in addition, on perceived ease of use.

The article "Investigating IT Faculty Resistance to Learning Management System Adoption Using Latent Variables in an Acceptance Technology Model" was published in 2015. Journal: ScientificWorldJournal.

In [10], the author built a model based on the TAM to examine technology acceptance among preservice teachers at a teacher training institute in Singapore. In his paper, the author highlights the success of the TAM in the business context and its limited application in educational contexts. He recalled that many studies had indicated that teachers do not use technology effectively. According to the author, this is due to the fact that teachers exert certain autonomy in their work. Teachers are also confronted with many variables such as computer self-efficacy, technological complexity, and facilitating conditions. Moreover, to evaluate the TAM in an educational context, the author assessed the extent to which the variables in the TAM predicted the technology acceptance among preservice teachers. Additionally, he considered the significance of the relationships between these external variables and those in the TAM. The resulting model showed that perceived usefulness appeared to be the strongest determinant of behavioral intention. On the other hand, these results revealed that the constructs of perceived usefulness, attitude toward computer use, and computer self-efficacy have a direct effect on preservice teachers' technology acceptance. In contrast, perceived ease of use, technological complexity, and facilitating conditions affect technology acceptance indirectly.

Other studies emphasize their research on the external variables [13] and their relationship with PEOU and PU. Among these studies are the following.

In [22], the research examined computer anxiety, computer self-efficacy, and perceived ease of use of an LMS. The study focused on the relationship between anxiety and PEOU and the role that mediating computer self-efficacy plays in that relationship. The study was conducted in an undergraduate online course setting spanning one year using an LMS as the target system. A survey instrument was used using three constructs: perceived ease of use, computer anxiety, and self-efficacy. The finding showed that computer self-efficacy plays an important role in mediating the impact of anxiety on PEOU of an LMS. The study results support the existence of a strong and significant relationship between anxiety and self-efficacy. It showed that as student anxiety increases, the perception of ease of use decreases and vice versa.

The article "Investigating IT Faculty Resistance to Learning Management System Adoption Using Latent Variables in an Acceptance Technology Model" was published in 2015. Journal: ScientificWorldJournal.

Furthermore, a study in [14] focused on the role of computer self-efficacy (CSE) and computer anxiety beliefs at the application level in the context of system acceptance and usage. The authors assessed the direct and indirect effects of application (CSE) and application anxiety on user's acceptance of an IS. The results showed that application self-efficacy has a strong impact on perceived ease of use and a significant one on perceived usefulness. According to the authors the results demonstrated that application-specific beliefs may offer better prediction of behavior than general beliefs.

In [23], the author conducted four studies. The work is part of an approach that combines the approaches of technology acceptance and a new space called “user experience.” In this new space, the author included variables such as computer anxiety, self-efficacy, prior experience, task complexity, perceived ease of use, and perceived usefulness. This research had two main goals: (1) examining the effect of the complexity level of tasks and of user mood on user experience and technology acceptance variables; (2) providing an integrative structural model that accounts for the contribution of instrumental and noninstrumental variables in the technology adoption process. The main results notably showed that usability perceptions are consistent with real usability level. In addition, it appears that affects and usability are particularly reactive variables to system usage.

Following the literature, over the years, research studies have identified numerous factors influencing the acceptance of technology with different external variables according to the context and culture in which this technology is used; there is no unique model that effectively applies to all contexts. Therefore, our study will investigate the resistance of our faculty members to using LMS through the usage of various constructs; this will be discussed next.

## 6. Research Design and Methodology

Based on the previous research that demonstrated the influence of usefulness and ease of use on the usage of e-learning [12, 20], we focused our study on the antecedents of these constructs. We will focus on (1) understanding the personal factors that influence LMS usefulness that plays an important role in the acceptance or rejection of technology and (2) examining the relationship among perceived usefulness (PU), perceived ease of use (PEOU), motivation, organizational support, and load anxiety (Figure 3).

### 6.1. Study Setting

King Saud University (KSU), similar to numerous other universities in the Middle East, introduced Blackboard as a learning management system in its institutions to serve as an online teaching and learning solution [24]. KSU has encouraged its faculty to employ Blackboard in their teaching practices. For example, the IT Department at the College of Computer and Information Sciences has been using Blackboard since 2010. The IT Department has used Blackboard as part of blended-learning practices, in which lectures are given in the traditional classroom setting while Blackboard is used to communicate and interact with students online. The version used is Blackboard Learn 9.1. The department had 50 lecturers and approximately 400 students during the Fall 2014 semester. The IT Department offers 30 courses each semester, and the academic calendar is divided into two semesters. The IT Department enrolls only female students, and all of the staff members, both academic and nonacademic, are female.

The article "Investigating IT Faculty Resistance to Learning Management System Adoption Using Latent Variables in an Acceptance Technology Model" was published in 2015. Journal: ScientificWorldJournal.

### 6.2. Data Collection Instrument

All teaching staff within the IT Department was invited to participate in this study. Data for this study were retrospectively collected from a survey instrument. Questions in the survey were selected among items previously published and validated in [5, 24, 25]. The survey consists of multiple-choice items, and five Likert*-*type scale questions were used to collect empirical data. In addition, open-ended questions were included in the survey to allow respondents to express their personal views. Questions were checked for clarity and appropriateness. The survey for faculty was designed to elicit responses about teaching and learning using the online learning management system of Blackboard. It comprised 4 sections: The first section collected characteristics of participants as well as experience in teaching, number of students in classes, and level of education. The second one covered questions to assess faculty perceptions of Blackboard in teaching in terms of motivation, organizational support, load anxiety, perceived usefulness, perceived ease of use, and actual use. The third section evaluated the features that were most often used and the degree of satisfaction in using these features. In the final section, faculty members were asked about the functionalities they desired in Blackboard. This survey also used binary (yes or no) questions to determine who is using Blackboard and their familiarity with the functions of Blackboard. The survey measured the relationships between the variables of perceived usefulness, perceived ease of use, motivation, load anxiety, perceptions of organizational support, and actual use.

### 6.3. Design of the Study

This is a regression study of faculty usage of LMS within the Information Technology (IT) Department, at the College of Computer and Information Sciences at King Saud University. A total of 50 faculty members work in the IT Department. Among them, we received 20 responses, which corresponded to a response rate of 40%. This corresponds to less than 50% of the total population providing feedback, but our sample size was sufficiently large. Among the 20 faculty participants, 16 instructors were using Blackboard and 4 were not using it during the Fall 2014 semester. All respondents were full-time female faculty. The majority of those faculty members who responded to the survey reported that they have used Blackboard while teaching 1–5 courses, and one faculty member had used it with more than 5 courses. The distribution of teaching experience was as follows: 1 faculty member had less than 1 year, 13 had 2–5 years, 5 had 6–10 years, and one faculty member had more than 10 years of traditional teaching experience. From these values, it can be seen that the surveyed faculty members were characterized by a large range of teaching experience.

The article "Investigating IT Faculty Resistance to Learning Management System Adoption Using Latent Variables in an Acceptance Technology Model" was published in 2015. Journal: ScientificWorldJournal.

### 6.4. Data Analysis Procedures

After the surveys were collected, the data were entered into SPSS Version 16 software to perform further analysis using Cronbach's alpha, regression, and descriptive statistics. Cronbach's alpha was used to measure internal consistency using the Reliability Analysis function in SPSS.

Data analysis was conducted in two stages. The first stage involved testing the various variables of perceived ease of use, perceived usefulness, motivation, load anxiety, and perceived organizational support for reliability using Cronbach's alpha. The second stage involved testing the dependent variables from the external variables using regression.

### 6.5. Findings and Analysis

The purpose of this study was to investigate the correspondence between faculty members' attitudes toward the use of Blackboard and their perceptions with regard to the constructs of motivation, load anxiety, perceived usefulness, perceived ease of use, organizational support, and actual use.

An internal consistency reliability test for the variables was conducted. The reliability test was performed in SPSS Version 16 using the Scale Reliability Analysis function.  Table 2 provides the results of this reliability testing.

Cronbach's alpha coefficients of the scales are presented in Table 2. All of the coefficients exceed 0.70. As a result, all of these four measures were deemed acceptable and valid. Actual use was not in our hypothesis. We assign just one question in the survey (Do you use Blackboard?) and that is why it received the lowest mean among other constructs. The other constructs include more items as shown in column 2 in Table 1.

Furthermore, we conducted correlation analysis among the variables as shown in Table 3. The benefit of the correlation matrix is to avoid multicollinearity among the variables and to build an accurate regression model. A high correlation value indicates redundancy among the input variables.

The article "Investigating IT Faculty Resistance to Learning Management System Adoption Using Latent Variables in an Acceptance Technology Model" was published in 2015. Journal: ScientificWorldJournal.

A standard regression analysis was performed between the dependent variable (one of each of the variables) and the independent variables (the remaining variables). Analysis was performed using SPSS regression as shown in Table 4. This table presents the result of simple regression of the interaction variables. It reports the model: the first column indicates the number of hypothesis, the second presents the dependent variables, and the third column shows the independent variables. Also included in this table are values for multiple correlation of *R* ^2^, *F*-values, regression coefficients, *P* values, and results of the testing of hypotheses.

We noticed from Table 3 that there is some correlation between support and motivation and between perceived usefulness and load anxiety, with values of 0.722 and 0.685, respectively. Nevertheless, none of the variables indicated high correlation values, as shown in the table, which signifies that there is no multicollinearity among the input variables. Therefore, all variables can be used while conducting the regression models, though the perceived ease of use has a negative correlation with all of the input variables. Therefore, the variable of perceived ease of use does not have an impact on the IT faculty members. This is because the IT faculties do not have a problem working with computers and are able to learn and adopt any software application easily. Hence, including or removing the perceived ease of use variable in the regression models would not have an impact on the results.

Regression analysis revealed as shown in Figure 4, for the first hypothesis (H1), that the dependent variable of motivation and other external variables (organizational support, perceived usefulness, and load anxiety) statistically significantly predicted attitude toward Blackboard, (*P* < 0.05) among the independent variables, excepting perceived ease of use. The regression model for motivation and ease of use had *P* > 0.05, which was not statistically significant. This supports the findings of Table 3, in which ease of use has negative correlations with all variables and does not have any impact on faculty attitude toward the usage of Blackboard.

Furthermore, we note that the highest *R* ^2^ value is 0.789, where the independent variables are all of the external inputs (load anxiety, PU, PEOU, and support). This could result because these input variables have a larger impact on the faculty perception of Blackboard more than the individual variable does. If an IT faculty member feels that LMS will reduce part of her teaching load, that it is useful and easy to use, and that support is available if needed, she will be more motivated to learn and use Blackboard.

The article "Investigating IT Faculty Resistance to Learning Management System Adoption Using Latent Variables in an Acceptance Technology Model" was published in 2015. Journal: ScientificWorldJournal.

Similarly, the second hypothesis (H2) models the dependent variable load anxiety with other variables (motivation, organization support, perceived usefulness, and perceived ease of use). The results were found to be statistically significantly predicting IT faculty members' attitudes toward LMS, with *P* < 0.05. But, organizational support and ease of use had *P* > 0.05, which were found not to statistically significantly affect the reduction in load anxiety.

IT faculty members are exposed to a variety of software applications and tools that can reduce their teaching load. Indeed, we have noticed from the faculty's feedback and survey responses that a large proportion of faculty members do not feel comfortable with Blackboard as an LMS. They believe that using Blackboard requires time and effort, which in turn increases their workloads. They recognized that Blackboard has some useful functions, but they perceived that this application is not intuitive to use.

Analogously, we examined the result of the third hypothesis (H3) where the dependent variable is organizational support and the independent variables are motivation, load anxiety, perceived usefulness, and perceived ease of use. We found a significant relationship between the organizational support and motivation and perceived usefulness. This could be due to the fact that the IT faculty members were observing the efforts from the e-learning deanship to support the usage of LMS. The deanship offers training during the year, answers faculty members' inquiries in a timely manner, and offers after-hours chat support. This kind of support makes LMS attractive to be used. However, IT faculty members still do not believe that this application will reduce their time and effort. We can see that the relationship between organizational support and load anxiety was found to be nonsignificant.

Finally, the last hypothesis (H4) related the dependent variable of perceived usefulness and the independent variables of motivation, organizational support, and perceived ease of use. We found the relationship between the LMS usefulness and the other independent variables to be significant.

From Table 4, we validate the constructs motivation, load anxiety, organizational support, PU, and PEOU. From faculty members' feedback, faculties acknowledged the usefulness of LMS in their teaching. However, they indicated some concerns with Blackboard, as shown below.

The article "Investigating IT Faculty Resistance to Learning Management System Adoption Using Latent Variables in an Acceptance Technology Model" was published in 2015. Journal: ScientificWorldJournal.

*Faculty Members' Comments*

*I find Blackboard useful and that it provides much functionality.*

*It is a very useful tool; however, it is slow and notifications are sometimes delayed.*

*My impression is that Blackboard is very useful especially in holding the course, gathering assignments, assigning grades through the grading center, and sending announcements.*

*It is good for announcements but usually takes a long time to notify students about contents.*

*It makes interaction with students easy.*

*I like it as a tool to replace blogs, especially it offers so much more such as an SMS tool …etc.*

From these comments, we can conclude that most faculty members surveyed who use Blackboard (11, i.e., 68%) found it useful as both a repository of course materials and a communication tool. The findings also indicated that some faculty members believe that several functionalities in Blackboard are complicated and that it takes a long time to complete a task.

#### 6.5.1. Level of Satisfaction with Blackboard Usage

Of the 20 faculty respondents, 16 were using Blackboard in the Fall 2014 semester, with the other 4 indicating that they were not using Blackboard to communicate with their students or to provide them with course materials.

The findings showed that most faculty respondents use Blackboard in the following ways to manage their courses: posting materials of their lectures (80%) as slides and assignments; communicating with their students through email (100%), SMS (65%), announcements (90%), and posting and calculating grades (55%). The most surprising aspect of the data was that nearly half (45%) of the faculty do not use it to deliver exams and quizzes and that the majority (55%) do not use it to conduct surveys. Interestingly, only 35% of the faculty respondents make use of the discussion board and assignment tool to assign, collect, and grade student work.

Further analysis shows that more than half (55%) of faculty members do not use reports to view lecture usage, 75% do not use Web 2.0 Tools, 40% do not use the calendar function, and 75% do not use chat or the virtual classroom.

Most faculty members indicated that they mainly use Blackboard to manage their courses. Interestingly, many instructors appreciated the features offered by Blackboard that enhance communication between them and their students, especially through email. However, other faculty respondents found that Blackboard is tedious, unclear, and difficult to use.

Table 5 shows that almost all 9 of the Blackboard features related to distance learning pedagogy have not been used by 75% of the faculty respondents. This is a surprising finding, considering the high level of technological ability possessed by these individuals. In fact, IT instructors most often use Blackboard as a storage venue for one-way dissemination of resources and material to students, similar to a blog.

The article "Investigating IT Faculty Resistance to Learning Management System Adoption Using Latent Variables in an Acceptance Technology Model" was published in 2015. Journal: ScientificWorldJournal.

*Features Desired to Be Added in Blackboard*. When asked what they would most like to be added as features in a future version of Blackboard (Table 5), faculty members preferred tools to ease the integration of online content, such as YouTube videos (60%); integration of email and calendar functions (60%); and interactive whiteboard function (45%).

These findings indicate an overall convergence between the desires and perceptions of Blackboard as a learning tool and its usage, expressed previously by faculty members. Faculty respondents felt that they were not able to design their courses in the way they wanted. They found that Blackboard lacks customization, while so many of them wish to have tools to build courses in ways to meet their specific needs. However, one faculty member reported that “in Blackboard Learn 9.1, the following tools are available as built in tools and are sufficient so far: YouTube video, Blog, Wikis, WileyPLUS. Lecture Capture, Recording & Interactive Whiteboard are embedded in Elluminate Live. News articles can be seen in the system Journal, Google Docs can be seen in the system KSU Drive.”

These findings show that faculty members are not necessarily aware of all functionalities available in Blackboard as shown in Table 6, which we believe is due to a lack of training and time invested to explore all functionalities available in Blackboard. In addition, slow Internet connections frustrated some instructors while they were using Blackboard, and many never tried to use it again.

## 7. Conclusion and Research Limitations

Learning management systems have been implemented in higher education in Saudi Arabia for many years. Nevertheless, teachers are not using it effectively, and sometimes this tool is not used at all. Our study intended to understand the personal factors influencing IT faculty members' acceptance or rejection of LMS. The researchers surveyed faculty perceptions of LMS as a teaching and a learning tool, respectively, including their level of satisfaction using LMS and an assessment of its degree of utilization in the IT Department. Data were collected via a survey distributed to all of the lecturers in the IT Department. Over 20 responses were received from faculty members, representing a response rate of 40%, which is an acceptable response rate for this kind of research within this field. Although this response rate is sufficiently large, the sample size remains a limitation of this study and does not allow the findings to be generalized. The study does not examine the comprehensive adaptation of the TAM to LMS usage. It focuses only on the latent variables, which are termed external variables in the TAM. This is due to a lack of data, since only a few faculty members who use LMS responded to the survey. Future studies should increase the scope and incorporate data from other departments, colleges, and disciplines within the university.

The article "Investigating IT Faculty Resistance to Learning Management System Adoption Using Latent Variables in an Acceptance Technology Model" was published in 2015. Journal: ScientificWorldJournal.

Similar to prior studies such as McFarland's research [6, 11], the findings of the present paper support that the adaptation of the TAM in a particular context would provide overall better results on latent variables and relationships among these variables. This study found many significant relationships between external variables such as motivation, anxiety, support, PEOU, and PU. Like previous studies [14, 19, 22] we found that motivation influences the PEOU and support influences motivation. These are the factors influencing the most LMS acceptance among IT faculties.

One interesting result of this study is that motivation, organizational support, and ease of use together are strong antecedents to the perceived usefulness construct of the TAM. Also, we found that the LMS ease of use alone has no impact on LMS usefulness. This can be explained by the fact that IT faculty members believe that they are able to manipulate any LMS or any other technological tool. Another interesting result is that motivation is impacted by the combination of organizational support, PEOU, load anxiety, and PU. This might indicate that the faculties are not willing to engage in new methods of teaching.

Findings from this study suggest that, by providing resources and fostering a supportive environment through the provision of time release to faculty members to manage their workload, leaders can reduce load anxiety and increase motivation and may consequently influence LMS use in the IT Department.

On the other hand, results from our survey showed that when faculty did use LMS, they did so to effectively manage their courses by providing materials to students and to send out announcements, emails, and sometimes SMS communications. Overall, this study shows that LMS is used essentially as an administrative tool rather than a teaching or learning tool.

The findings from this study have been determined to be consistent with the findings of several related studies on perceptions, usage, and attitudes of faculty members toward LMS such as Blackboard [26]. Most faculty members are not using LMS to its full potential. We can see from the findings above that posting announcements and materials and emailing are the most commonly used features by faculty. These functions have a high rate of reported satisfaction among the faculty who use them, while other important functions are eliminated. We suggest that faculties enhance their teaching style with the adopting of LMS.

The article "Investigating IT Faculty Resistance to Learning Management System Adoption Using Latent Variables in an Acceptance Technology Model" was published in 2015. Journal: ScientificWorldJournal.

## Figures and Tables

**Figure 1:** Technology acceptance model of Davis [5].

**Figure 2:** McFarland and Hamilton model [6].

**Figure 3:** Theoretical relationships between different constructs impacting LMS usage.

**Figure 4:** Research results of latent variables relationship.

**Table 1:** Variables.

Variables	Definition	Previous studies
Motivation	Four items measuring faculty motivation to use LMS as e-learning platform.	[9, 11]

Anxiety	Four items measuring fear of faculties to increase workload when using LMS.	[6, 8, 14]

Organizational support	Two items assessing universities resource support.	[6, 9, 10]

Perceived ease of use	Five items measuring the degree to which a person believes the LMS usage will be free of effort.	[5, 6, 8, 13]

Perceived usefulness	Six items measuring the degree to which a person believes the LMS usage will enhance job performance.	[5, 6, 8, 13]

**Table 2:** Internal consistency reliability testing.

Construct/variable	Total items	Means	Standard deviation	Cronbach's alpha
Motivation	4	3.30	0.733	0.756
Load anxiety	4	3.00	0.562	0.766
Support	2	2.35	0.587	0.772
PU	5	3.40	0.821	0.753
PEOU	6	3.35	0.489	0.798
Actual use	1	1.80	0.410	0.776

**Table 3:** Correlation matrix.

	Motivation	Load anxiety	Support	PU	PEOU	Actual use
Motivation	1.00					
Load anxiety	0.511	1.00				
Support	0.722	0.319	1.00			
Perceived usefulness (PU)	0.753	0.685	0.459	1.00		
Perceived ease of use (PEOU)	−0.308	−0.383	−0.449	−0.498	1.00	
Actual use	0.385	0.228	0.087	0.563	0.105	1.00

**Table 4:** Direct effect between independent constructs.

Hypothesis	Dependent variables	Independent variables	*R* ^2^	*F*-value	*β*	*P* value	Validation
H1	Motivation	Load anxiety	0.261	6.37	0.667	0.021	Significant
		Support	0.521	0.000	0.901	0.0	Significant
		Perceived usefulness	0.566	23.5	0.672	0.0	Significant
		Anxiety + support + PU + PEOU	0.789	14.0	For each	0.0	Significant
		Ease of use	0.095	1.89	−0.462	0.186	Not significant

H2	Load anxiety	*Motivation*	0.261	6.372	0.392	0.021	Significant
		Perceived usefulness	0.469	15.882	1.406	0.001	Significant
		Support	0.102	2.04	0.305	0.170	Not significant
		Ease of use	0.147	3.09	−1.758	0.096	Not significant

H3	Organization support	Motivation	0.521	19.581	0.578	0.000	Significant
		Load anxiety	0.21	4.796	0.328	0.09	Not significant
		Perceived usefulness	0.201	4.54	−0.538	0.042	Significant
		Ease of use	0.521	19.581	0.578	0.047	Significant

H4	Perceived usefulness	*Motivation + support + ease of use*	0.699	12.365		0.000	Significant
		*Motivation + ease of use*	0.645	15.418		0.000	Significant

The article "Investigating IT Faculty Resistance to Learning Management System Adoption Using Latent Variables in an Acceptance Technology Model" was published in 2015. Journal: ScientificWorldJournal.

**Table 5:** Faculty usage of Blackboard features.

Blackboard features	HS + MS	SS	NS	NU
Posting: documents, PowerPoint, and PDFs	65%	5%	20%	10%
Emailing students & colleagues	80%	5%	5%	0%
SMS tool	30%	15%	10%	35%
Posting course announcements	70%	10%	5%	10%
Delivering online exams and quizzes	20%	20%	5%	45%
Delivering online surveys	15%	5%	15%	55%
Posting and calculating grades	20%	10%	10%	50%
Online discussion board	10%	10%	5%	65%
Assignment tool for assigning, collecting, and grading student work	15%	5%	5%	65%
Reports to view information about course usage and activity	15%	15%	5%	55%
Web 2.0 Tools (blogs, wikis, podcasts, and private journals)	10%	0%	5%	75%
Blackboard Learn calendar	5%	0%	10%	40%
Blackboard Learn chat	5%	0%	10%	75%
Blackboard Learn virtual classroom (*Elluminate Live!*)	5%	5%	5%	75%

**Table 6:** New features requested by faculty.

New features requested by faculty	*N* (total)	
e-portfolios	2	10%
Ability to post your work to “the outside world” (give it a public URL)	7	35%
Personal profiles (Facebook-style)	1	5%
Built-in tools to integrate YouTube videos, Flickr photos, news articles, blog posts, and Google	12	60%
Docs. and other web content integrated into online courses	0	0%
Notifications to your Facebook, Twitter, or other social media	5	25%
Lecture capture & recording	6	30%
Interactive whiteboard	9	45%
Integration with online email and calendar	12	60%
Others	1	5%
